The article "Retrieval-Based Factorization Machines for Human Click Behavior Prediction" was published in 2022. Journal: Comput Intell Neurosci.

# Retrieval-Based Factorization Machines for Human Click Behavior Prediction

**DOI:** 10.1155/2022/1105048

**Published:** 2022-11-18

**Authors:** Yu Tang, Sheng Wang, Yuancai Huang, Xiaokai Zhao, Weinan Zhao, Yitao Duan, Xu Wang

**Affiliations:** ^1^Beihang University, Beijing, China; ^2^Beijing Institute of Space Launch Technology, Beijing, China; ^3^Kuaishou Inc, Beijing, China; ^4^Netease Youdao Information Technology Ltd, Beijing, China; ^5^Zhongguancun Laboratory, Beijing, China

## Abstract

Human click behavior prediction is crucial for recommendation scenarios such as online commodity or advertisement recommendation, as it is helpful to improve the quality and user satisfaction of services. In recommender systems, the concept of click-through rate (CTR) is used to estimate the probability that a user will click on a recommended candidate. Many methods have been proposed to predict CTR and achieved good results. However, they usually optimize the parameters through a global objective function such as minimizing logloss or root mean square error (RMSE) for all training samples. Obviously, they intend to capture global knowledge of user click behavior but ignore local information. In this work, we propose a novel approach of retrieval-based factorization machines (RFM) for CTR prediction, which can effectively predict CTR by combining global knowledge which is learned from the FM method with the neighbor-based local information. We also leverage the clustering technique to partition the large training set into multiple small regions for efficient retrieval of neighbors. We evaluate our RFM model on three public datasets. The experimental results show that RFM performs better than other models in metrics of RMSE, area under ROC (AUC), and accuracy. Moreover, it is efficient because of the small number of model parameters.

## 1. Introduction

Human click behavior prediction is important for recommendation scenarios in many online commercial services. In those scenarios, recommended items such as online commodities, advertisements, and videos are often displayed to end users for clicking. Service providers expect more clicks from end users on the recommended items because that means more revenue from advertisers, and it is helpful to improve user satisfaction [1]. Therefore, it is crucial to accurately predict the click-through rate (CTR) for these recommendation scenarios [1, 2], as CTR can indicate the probability that a user will click on a recommended candidate.

CTR prediction relies on the analysis of historical click behavior data. The click behavior data include mostly discrete and categorical features, such as user gender, user id, commodity category, commodity id, and other location or demographic information. Thus, it can be highly sparse and has complicated feature interactions. Generalized linear models are applied to predict CTR including logistic regression [3] and support vector machines [4], which have difficulties to capture high-order feature interactions. Then, factorization machines (FM) [5] were proposed to model order-2 feature interactions by the inner product of latent vectors between different features and achieve very promising performance. Based on FM, field-aware factorization machines (FFM) [6] divide features with different fields and extend FM with additional field-aware feature interactions. In addition, high-order factorization machines (HOFM) [7] were presented to model high-order (more than 2) feature interactions but are limited by high training complexity.

The article "Retrieval-Based Factorization Machines for Human Click Behavior Prediction" was published in 2022. Journal: Comput Intell Neurosci.

Recently, deep learning has made massive strides in many research areas obtaining state of art performance in computer vision [8], natural language processing [9], and many other domains [10–12]. In order to learn sophisticated feature interactions, deep neural networks were recently proposed to predict CTR [13–17]. Based on the feature embedding, firstly, the features are represented by one-hot vectors and embedded in low-dimensional dense vector. Wide&Deep [13] feeds these feature embeddings to a combination of linear model and DNN to achieve both low-order and high-order feature interactions. DeepCross [14] uses a multilayered residual network to prevent gradient explosion and vanishing problems when the depth of the network increases. DeepFM [15] combines FM and DNN through sharing feature embedding vectors. NFM [16] obtains second-order feature interaction vectors by FM and feeds them into fully connected layers. AFM [17] applies an attention mechanism to second-order interaction vectors, which model the importance of different interactions. These deep learning methods can represent low-order and high-order feature interactions well and thus obtain good performance for CTR prediction.

However, these methods above [5, 13–17], including FM and FM-based neural models, usually train the models and optimize the parameters through a global objective function, such as minimizing logloss or mean square error for all training samples. Obviously, they intend to capture global knowledge of user click behavior but ignore local information such as the most similar samples. The local information has been considered in collaborative filtering based on the memory network [18, 19]. But these methods only utilize user-item interaction information. In the CTR prediction task, there are some content and contextual information that they miss such as user demographics, time, and locations. Also, the training set is usually very large, and the local information from the training set changes for different testing samples; thus, efficiency is critical for retrieving such local information.

The article "Retrieval-Based Factorization Machines for Human Click Behavior Prediction" was published in 2022. Journal: Comput Intell Neurosci.

In this work, we propose a novel approach of retrieval-based factorization machines (namely RFM) for CTR prediction, which enhances FM by retrieving similar samples from the training set as the neighbor-based local information. Specifically, firstly, we train a standard FM model by the feature embedding and the second-order feature interaction embedding. Based on the sample representation of the second-order feature interaction embedding, we can retrieve similar samples from the training set for one given testing sample. In order to improve the efficiency of retrieving similar samples from the large training set, we preprocess to partition the training set into multiple small regions by the clustering algorithm K-means. During the testing phase, we get the most similar region by computing the similarity between the testing sample and the center vectors of all regions. Then, we retrieve the most similar samples as neighbors from the region and finally enhance the FM model by fusing the neighbor-based local information and the original FM output via the weighted sum. We conduct extensive experiments on three public datasets to evaluate our RFM method. The experimental results show that RFM outperforms FM and existing studies such as HOFM [7] and deep learning models including DeepCross [14], Wide&Deep [13], and DeepFM [15]. In addition, RFM has the same number of trainable parameters with FM, which is much smaller than those of other studies. Therefore, RFM is an efficient and effective approach for CTR prediction. Compared with the black box of deep neural models, RFM is also more explicable due to its simple and easily understood architecture.

In summary, this paper makes the following contributions:

- We propose a novel approach of retrieval-based factorization machines (RFM) for CTR prediction, which can enhance FM by the neighbor-based local information
- We use the clustering technique to partition the large training set into multiple small regions for efficient retrieval of similar samples
- We conduct extensive experiments to evaluate RFM on three public datasets, and the experimental results show that RFM performs better than existing models and is efficient due to the smallest number of model parameters

The remainder of this paper is organized as follows.

Firstly, we discuss related works in Section 2.  Section 3 describes the embedding methods for FM. Afterwards, we describe the details of our approach in Section 4.  Section 5 describes datasets, evaluation procedures, and evaluation results. Finally, we conclude our work in Section 6.

The article "Retrieval-Based Factorization Machines for Human Click Behavior Prediction" was published in 2022. Journal: Comput Intell Neurosci.

## 2. Related Work

CTR prediction is an important task of the recommendation domain [1, 2]. In this section, we discuss the related work about traditional machine learning methods, deep learning models, and memory-based models in the recommender systems.

For CTR prediction, some traditional machine learning methods have been proposed in the early stage, such as support vector machine [4], Bayesian model [20], tensor-based model [21], linear regression [22], and decision tree [3]. After that, factorization machine [5] (FM) is proposed. It projects each feature into a latent vector and captures the second-order feature interaction information. Field-aware factorization [6] (FFM) and high-order factorization machine [7] (HOFM) are the enhanced factorization machine. FFM adopts field to FM, and HOFM models high-order (more than (2)) feature interactions. For the general recommendation scene, collaborative filtering [23] (CF) is a traditional and fundamental method. Matrix factorization [24] (MF) which projects each user and item into a common low-dimensional space capturing latent relations is a famous method based on CF.

With the wide use of deep learning in various fields, many deep learning models have been proposed for CTR prediction [25–29]. Their bottom-level structure is an embedding layer mapping categorical variables to lower-dimension dense vectors. DeepFM [15] combines FM and DNN through sharing embedding parameters to represent low-order and high-order feature interactions. AFM [17] and NFM [16] are based on second-order feature interaction vectors. NFM feeds these vectors into fully connected layers, and AFM applies an attention mechanism to these vectors to model the importance of different interactions. HoAFM [30] encodes high-order feature interactions into feature representations in an explicit manner. Besides, the convolutional click prediction model [25] uses a convolution neural network to process a matrix consisting of embedding vectors, and deep&cross network [26] combines cross network and deep network. Its cross network causes the degree of cross features to grow with layer depth. Product-based neural network [27, 28] introduces a product layer to capture interaction information. Recurrent neural network for sequential click prediction [29], deep interest network [31], and deep interest evolution network [32] take advantage of users' history click behaviors sequence to predict CTR. Convolution neural network for CTR prediction in display advertisement [33] combines convolution neural network processing raw images in display and general deep network. Several deep learning methods are proposed in recommendation tasks. They are used for recommending video [34], music [35], and movies [36] improving collaborative filtering via deep learning. Generalized matrix factorization [37] and neural network matrix factorization [38] improve MF via deep learning.

The article "Retrieval-Based Factorization Machines for Human Click Behavior Prediction" was published in 2022. Journal: Comput Intell Neurosci.

Compared with the traditional machine learning methods and deep learning models above for CTR prediction, we consider the neighbor-based local information to enhance the FM method.

In the field of collaborative filtering, there are also some studies [18, 19, 39] that introduce neighbor-based local information [40] to improve their methods based on the memory network [9, 41], including collaborative memory network [18], multirelational memory network [19], and collaborative session-based recommendation machine [39]. Their main idea is fusing a memory component and neural attention mechanism as the neighborhood component. Also, knowledge enhances the sequential recommendation [42] through integrating RNN-based networks with key-value memory network [43]. However, they usually only consider specific feature interactions such as the user and item feature interaction, and our RFM method considers the content and contextual information and leverages the region partition to further improve the efficiency and performance.

Our earlier work entitled “Retrieval-based Factorization Machines for CTR Prediction” in WISE 2021 presents the main idea of RFM. In this extended paper, we demonstrate more details on the design of RFM, including dropout, batch normalization, and the selection strategy on top-k neighbors. Besides, we analyze our RFM model by comparing RFM with existing FM-based neural models and collaborative filtering methods based on the memory network in the aspects of complexity and the cold-start problem analysis. Moreover, we evaluate the impact of more hyperparameters including the embedding size, the number of similar samples, and the similarity threshold via conducting extensive experiments. Finally, we present a more detailed analysis of related work.

## 3. Background

In this section, we provide the background of FM and FM-based neural models, including the feature embedding and second-order feature interaction embedding.

### 3.1. Feature Embedding

For the task of CTR prediction, the features of historical click behavior data typically have categorical fields (e.g., gender, commodity categories) and continuous fields after discretization (e.g., cost, age). These fields are usually converted to a set of binary features via one-hot encoding, making the original feature vectors highly sparse.

The article "Retrieval-Based Factorization Machines for Human Click Behavior Prediction" was published in 2022. Journal: Comput Intell Neurosci.

One common practice is encoding the sparse feature vectors to low-dimensional dense vectors by feature embedding. Given one sample *x* with *n* fields and the *i*-th field vector *x*_*i*_(1 ≤ *i* ≤ *n*) via one-hot encoding. We map each field vector *x*_*i*_ to an embedding vector *v*_*i*_ ∈ *R*^*d*^ by

(1) $$\begin{array}{c} v_{i}={W_{e}}^{⊤}x_{i},i\in \left[1,n\right]\text{,} \end{array}$$

where *W*_*e*_ is the latent factor matrix that can be learned in one end-to-end manner, and *d* is the embedding size. Then, we denote the output of the feature embedding as follows:

(2) $$\begin{array}{c} V\left(x\right)=\left[v_{1},v_{2},\ldots ,v_{n}\right]\text{.} \end{array}$$

The feature embedding technique has been adopted in Wide&Deep [13], DeepFM [15], and DeepCross [14] to reduce the data sparsity. Such embeddings are treated as the input of their models.

### 3.2. Second-Order Feature Interaction Embedding

Besides the (first-order) feature embedding described above, the second-order feature interaction embedding is also widely used in FM-based neural models including NFM [16] and AFM [17]. These methods feed feature embedding *V*(*x*) into the biinteraction layer [16] and obtain the second-order feature interaction embedding as follows:

(3) $$\begin{array}{c} S\left(x\right)=\overset{n}{\underset{i=1}{\sum }}\overset{n}{\underset{j=i+1}{\sum }}x_{i}\nu_{i}⊙x_{j}\nu_{j}\text{,} \end{array}$$

where ⊙ denotes the element-wise product of two vectors, that is, (*v*_*i*_⊙*v*_*j*_)_*k*_=*v*_*ik*_*v*_*jk*_.

Compared with the feature embedding, the second-order feature interaction embedding can capture more knowledge of user click behaviors and has been proven to be more effective in CTR prediction [16, 17]. Thus, we adopt the second-order feature interaction embedding in this work.

## 4. Retrieval-Based Factorization Machines

In this section, we describe the approach of retrieval-based factorization machines (RFM) for CTR prediction, which can enhance FM with retrieved neighbor-based local information. As shown in Figure 1, firstly, we train a standard FM to obtain the global knowledge of user click behaviors (Section 3.2) and obtain the second-order feature interaction embeddings; secondly, we partition the training set to different regions by a clustering algorithm based on the second-order feature interaction embeddings (Section 4.2). Such regions can be used to efficiently retrieve similar samples from testing samples and get the neighbor-based local information (Section 4.3). Finally, we enhance FM for predicting CTR by fusing the global and local information (Section 4.4).

### 4.1. Factorization Machines

Similar to existing FM-based neural models [15–17] for CTR prediction, firstly, we train the feature embedding layer and the second-order feature interaction embedding layer. Instead of feeding the embeddings to upper neural models, we use them to build a standard FM model, as described in Section 3. Given the sample *x* as input, the predicted CTR is

(4) $$\begin{array}{c} {\hat{y}}_{g}\left(x\right)=b+\overset{n}{\underset{i=1}{\sum }}w_{i}x_{i}+\overset{d}{\underset{i=1}{\sum }}S{\left(x\right)}_{i}, \end{array}$$

where *w*_*i*_ represents the weights of field vectors, and *b* is the bias. The first and second terms are the linear part, which reflects the importance of first-order features. The third term represents the impact of the second-order feature interactions. Similar to FM [5], the third term can be reformulated by

(5) $$\begin{array}{c} \overset{d}{\underset{i=1}{\sum }}S{\left(x\right)}_{i}=\frac{1}{2}\cdot \overset{d}{\underset{f=1}{\sum }}\left({\left(\overset{n}{\underset{i=1}{\sum }}v_{if}x_{i}\right)}^{2}-\overset{n}{\underset{i=1}{\sum }}v_{if}^{2}x_{i}^{2}\right), \end{array}$$

which not only reduces the computation complexity to *O*(n d) but also can be translated to matrix operation, which can be accelerated by GPU.

The article "Retrieval-Based Factorization Machines for Human Click Behavior Prediction" was published in 2022. Journal: Comput Intell Neurosci.

Based on (4), existing works [15–17] usually train FM and optimize model parameters through a global objective function such as minimizing the global mean square error. Thus, obviously, FM intends to capture the global knowledge of user click behaviors in the training set but ignores the local information such as the most similar samples in the training set.

### 4.2. Region Partition

In order to obtain the local information of one given sample in the testing set, we try to retrieve the similar samples from the training set as its neighbors based on the second-order feature interaction embedding (section 3.2). However, the training set is often very large. Thus, it will incur much overhead to directly compute the similarities among the training set. To solve this problem, as preprocessing, we adopt K-means [44], a classical clustering algorithm, to partition the training set into multiple regions. Then, we leverage these regions to accelerate the retrieval of similar samples. The clustering algorithm runs only once, and its result can be used for all testing samples.

Specifically, given all samples *X* in the training set and the *i*-th sample *X*_*i*_, we get the representation of sample *X*_*i*_ based on the second-order feature interaction embedding by

(6) $$\begin{array}{c} {emb}_{i}=BN\left(S\left(X_{i}\right)\right)\text{,} \end{array}$$

where we adopt batch normalization (BN) [45] to normalize the embedding *S*(*X*_*i*_) and keep the distribution of emb_*i*_ consistent. Similar to (5), we reformulate *S*(*X*_*i*_) to improve the efficiency as follows:

(7) $$\begin{array}{c} S\left(X_{i}\right)=\frac{1}{2}\cdot \left({\left(\overset{n}{\underset{j=1}{\sum }}v_{j}X_{ij}\right)}^{2}-\overset{n}{\underset{j=1}{\sum }}v_{j}^{2}X_{ij}^{2}\right)\text{.} \end{array}$$

Based on the representation emb_*i*_, we adopt the popular clustering algorithm *K*-means [44] to partition all the samples in the training set to multiple regions. In the K-means algorithm, we compute the Euclidean distance between sample representations and obtain *k* regions as follows:

(8) $$\begin{array}{c} C=\left\{c_{1},c_{2},\ldots ,c_{k}\right\},U=\left\{u_{1},u_{2},\ldots ,u_{k}\right\}\\ s.t.\;c_{1}\cap c_{2}\cap \ldots \cap c_{k}=\emptyset ,c_{1}\cup c_{2}\cup \ldots \cup c_{k}=X, \end{array}$$

where *C* is the set of the sample regions, and *U* is the set of center vectors for different regions. Each sample in the region *c*_*i*_ is a tuple described as (*x*, *y*), where *x* is the emb_*i*_ vector representation, and *y* is the corresponding label. All the regions are disjoint, and their union is the whole training set. *k* is the number of regions and can be manually tuned.

The article "Retrieval-Based Factorization Machines for Human Click Behavior Prediction" was published in 2022. Journal: Comput Intell Neurosci.

After clustering, we partition all samples in the training set to *k* regions, and the center vectors *u*_*i*_ can represent the characteristics of all samples in one same region. We find the most similar region based on the center vectors and then retrieve the similar samples from the region. In this way, we reduce the computation complexity of retrieving similar samples among the whole training set.

Intuitively, our retrieved similar samples may not be the most similar ones from the whole training set and probably decrease the performance since we adopt the center vectors to represent all the samples of same regions. However, the clustering technique reveals the intrinsic nature and regularity [46, 47] in the training set, and the most similar samples retrieved from the same region may contain more effective and generalizable information than those from the whole training set. That is, why partitioning into more than one region may lead to better performance than not partitioning, which is observed in our experiments (section 5.7.1). Therefore, such partitioning not only increases the retrieval efficiency but also improves the performance.

### 4.3. Neighbor-Based Local Information

Based on the disjoint regions of the training set, we introduce an efficient approach to retrieve similar samples as the neighbors for one given testing sample. Instead of computing the most similar samples directly from the large training set, we get the most similar sample region by calculating the similarity between the center vectors of regions and the representation of the testing sample. Then, we retrieve the most similar samples as neighbors from the region. Finally, we choose top-*t*(*t* ≥ 1) neighbors with the most similarities to capture more local information and adopt the similarity threshold to filter out possible noisy neighbors.

The article "Retrieval-Based Factorization Machines for Human Click Behavior Prediction" was published in 2022. Journal: Comput Intell Neurosci.

Specifically, we first measure the similarity between sample *X*_*i*_ and *X*_*j*_ based on their representations by

(9) $$\begin{array}{c} sim\left({emb}_{i},{emb}_{j}\right)=\frac{1}{1+{dist}_{ed}\left({emb}_{i},{emb}_{j}\right)}\\ {dist}_{ed}\left({emb}_{i},{emb}_{j}\right)={\left\|{emb}_{i}-{emb}_{j}\right\|}_{2}, \end{array}$$

where dist_*ed*_(emb_*i*_, emb_*j*_) represents the function computing Euclidean distance between emb_*i*_ and emb_*j*_. The smaller the distance between two samples is, the higher the similarity between them is. Then, we can get the most similar sample region as follows:

(10) $$\begin{array}{c} g=\arg\max_{j\in \left[1,k\right]}\;sim\left(u_{j},{emb}_{0}\right)\text{,} \end{array}$$

where emb_0_ is the representation of the given sample, and *g* is the index of the most similar sample region in the region set *C*.

We finally show how to retrieve top-*t* neighbors with the similarity threshold *r* from the region *c*_*g*_ in Algorithm 1.

As shown in Algorithm 1, the threshold *r* is used to filter out possible noisy neighbors (line 2). The output *N* is a list of tuples (sim, *y*) containing the similarity and labels of neighbors. The function selectTop in line 8 selects top-*t* similar samples from neighbors, and it will be discussed in section 4.5.4. Obviously, the more similar the neighbors are, the more sufficient the information provided by neighbors will be. The high similarity threshold will filter out some useful neighbor-based information. On the contrary, the low similarity threshold will introduce noise that makes side effect on prediction. Additionally, the number of selected neighbors *t* also influences the performance. The impact of the similarity threshold *r* and the neighbor number *t* will be discussed in Section 5.

Compared with the global knowledge from all the training sets, the retrieved neighbors are only a small subset. But they usually represent the common knowledge of these similar click behaviors, which can be treated as the local information of the given testing sample.

### 4.4. Enhancing FM with Local Information

To improve the FM model, we fuse the retrieved neighbor-based local information *N* and the global information ${\hat{y}}_{g}\left(x\right)$ provided in section 4.1.

The article "Retrieval-Based Factorization Machines for Human Click Behavior Prediction" was published in 2022. Journal: Comput Intell Neurosci.

Specifically, we add the weighted sum of neighbor information to the original FM output and normalize the result as follows:

(11) $$\begin{array}{c} \hat{y}\left(x\right)=\frac{{\hat{y}}_{g}\left(x\right)+\beta \sum_{i=1}^{t}y_{i}\cdot {sim}_{i}}{1+\beta \sum_{i=1}^{t}{sim}_{i}}, \end{array}$$

where *t* is the number of retrieved neighbors, and *y*_*i*_ and sim_*i*_ are the labels and similarities of neighbors, respectively. For balancing the global and the local effect, we add a factor *β* to control the effect of the local information, which can be manually tuned. Since the range of similarities between the given sample and other samples in the training set is between 0 and 1, thus we can also change *β* from 0 to 1. If the neighbor similarities are relatively small, we can turn up *β*. On the contrary, we turn down *β* to consider less local information.

### 4.5. Training and Testing

Since the joint training for all the samples in the training set and their corresponding neighbors are very expensive, we only train a standard FM model and fuse neighbor-based local information and the original FM output during testing. In the training phase, we use one global objective function to update trainable parameters for standard FM. Then, we can obtain the second-order feature interaction embeddings for representing samples and region partition. Finally, during the testing phase, we retrieve the neighbors and enhance FM by fusing the original FM output and the neighbor-based local information.

#### 4.5.1. Objective Function

FM can be applied to various prediction tasks, including regression, classification, and ranking. In our task of CTR prediction, we adopt the widely used objective function square loss:

(12) $$\begin{array}{c} L_{reg}=\underset{x\in X}{\sum }{\left({\hat{y}}_{g}\left(x\right)-y\left(x\right)\right)}^{2}, \end{array}$$

where *X* represents the set of instances for training, and *y*(*x*) represents the target of instance *x*.

#### 4.5.2. Dropout

We use emb_*i*_ to represent any sample *X*_*i*_, and its dimension is *d*. If we assign a large value to *d*, it may lead to overfitting. In order to alleviate this problem, we introduce the technique of dropout [48] for training. Dropout is a regularization technique to avoid overfitting. Its idea is to drop neurons randomly during training. Only part of the model parameters which contribute to the prediction of ${\hat{y}}_{g}\left(x\right)$ will be updated in each iteration. In the testing phase, dropout is disabled, and all parameters are used for estimating ${\hat{y}}_{g}\left(x\right)$.

#### 4.5.3. Batch Normalization

As described in Section 4.2, we normalize the second-order feature interactions embedding vectors through batch normalization [45] to keep the distribution of *emb*_*i*_ consistent. BN normalizes inputs to a zero-mean unit-variance Gaussian distribution. Formally, given an input vector *X*_*i*_ ∈ *R*^*d*^ and all input vectors to the layer of the mini-batch be *B*={*X*_*i*_}, the BN normalizes *X*_*i*_ as follows:

(13) $$\begin{array}{c} BN\left(X_{i}\right)=\gamma ⊙\left(\frac{X_{i}-\mu_{B}}{\sigma_{B}}\right)+\beta , \end{array}$$

where *μ*_*B*_, *σ*_*B*_^2^ denote the mini-batch mean and variance separately, and *γ* and *β* are trainable parameters to scale and shift normalized value to restore the representation power of the model. BN is applied in both the training and testing phases in our RFM model.

The article "Retrieval-Based Factorization Machines for Human Click Behavior Prediction" was published in 2022. Journal: Comput Intell Neurosci.

#### 4.5.4. Selection of Top-*t* Neighbors

In the testing phase, we fuse neighbor-based local information and the original FM output online. The bottleneck is how to efficiently select top-*t* neighbors from the most similar sample region. We briefly discuss three alternative methods. The first is sorting neighbors by similarity in the descending order and selecting the first *t* neighbors. The second is quick selection by adopting the idea of divide and conquer; that is, we swap samples by comparing pivots in subinterval recursively until the length of the subinterval is equal to *t*. The elements in the subinterval are the results. The third is using the priority queue implemented by the heap. We can build a priority queue with *t* size, push neighbors to the queue, and the queue will pop neighbors with small similarity dynamically. When going through all neighbors, the neighbors in the priority queue are the results. In this work, we adopt the quick sort algorithm to select the top-*t* neighbors for good efficiency.

### 4.6. Comparison with Existing Models

We compare our RFM model with existing FM-based neural models and collaborative filtering methods based on the memory network in the aspects of complexity and the cold-start problem [49].

#### 4.6.1. Complexity Analysis

The scale of trainable parameters of our RFM model is much smaller than neural models, including NFM [16], DeepFM [15], Wide&Deep [13]. The parameters' number of the embedding layers is *n* × *d*, and the linear weights parameters in global output are *n*. The bias in global output and two parameters in batch normalization are constant; thus, we omit them. In the testing phase, we need to store neighbors retrieved from similar samples, which take *t* × *d* storage units. Thus, the space complexity of our model is *O*((*n*+*t*)*d*+*n*). The deep learning models mentioned above have not only embedding layers but also plenty of fully connected layers. Thus, the number of trainable parameters in these models increases exponentially with the number of layers.

The article "Retrieval-Based Factorization Machines for Human Click Behavior Prediction" was published in 2022. Journal: Comput Intell Neurosci.

In computation complexity, we reduce the complexity of computing global output ${\hat{y}}_{g}\left(x\right)$ to *O*(*n* *d*). In the testing phase, we compute the similarity between a given sample and samples from the most similar region in *O*(*dN*), where *N* is the number of samples in the region. After that, we select the top-*t* neighbors in *O*(*N* log *N*). The computation complexity of our model is *O*((*n*+*N*)*d*+*N* log *N*). In the deep learning method, the complexity of computation also increases exponentially with the number of layers.

#### 4.6.2. Cold-Start

It is difficult to conduct personalized recommendations without enough historical data of users (i.e., the cold-start problem [49]), which is common in recommender systems and has been studied for a long time [50–52].

Existing memory-based models including collaborative memory network [18] and multirelational memory network [19] also leverage the idea of fusing global information and local information, but both models only use the user and item interaction information. When a new user comes, they cannot map it to an effective vector due to the lack of historical click data for the user. By contrast, our RFM model takes full advantage of user demographics, which can be easily obtained such as the registry information and the contextual information like the time and location. Thus, it can capture effective feature interaction information and neighbor-based local information for CTR prediction. In this way, our RFM model can adapt to the cold-start scenario better.

## 5. Evaluation

In this section, we conduct extensive experiments to evaluate our RFM approach on three public datasets. We first show the superior performance of RFM and analyze the effectiveness of neighbor-based local information. We also investigate the impact of hyperparameters, in particular, the number of regions in partitioning (Section 4.2) and neighbor-based local information (Section 4.3).

### 5.1. Data Set Description

We evaluate RFM on three public datasets: Frappe [53], MovieLens (https://grouplens.org/datasets/movielens/latest/), and Criteo (https://labs.criteo.com/2014/02/download-kaggle-display-advertising-challenge-dataset/), which are widely used in CTR prediction.

- Frappe Dataset: This dataset is often used in the context-aware recommendation. It contains 96,203 app usage logs of users under different contexts. It contains eight context variables except for user ID and app ID, which are all categorical, including weather, city, and daytime. We convert each log (user ID, app ID, and context variables) to a feature vector via one-hot encoding.
- MovieLens Dataset: This dataset has been used for personalized tag recommendation. It contains 668,953 tag applications of users on movies. We also convert each tag application (user ID, movie ID, and tag) to a feature vector.
- Criteo Dataset: This dataset includes 45 million users' click records and has 13 continuous features and 26 categorical features. It has been widely used for the display advertising challenges. We discretize the continuous features and convert them by using a tool provided in the Kaggle challenge (https://github.com/ycjuan/kaggle-2014-criteo).

The article "Retrieval-Based Factorization Machines for Human Click Behavior Prediction" was published in 2022. Journal: Comput Intell Neurosci.

For Frappe and MovieLens, if one log is assigned a label of value 1, we treat it as “clicked” which means that the user has used the app under the context or applied the tag on the movie. We randomly select the logs representing that the user does not use the app or the tag is not applied on the movie as negative samples and assign −1 to their labels. Finally, we get 288,609 and 2,006,859 samples, respectively. We randomly split each dataset into three parts: 70% for training, 20% for validation, and 10% for testing. We use the validation set for tuning hyperparameters and the testing set for performance comparison. For Criteo, we make random sampling and get 458,406 samples. We also split them into training, validation, and testing parts using the same ratio.

### 5.2. Evaluation Metrics

We adopt root mean square error (RMSE), area under ROC (AUC), and accuracy to evaluate the performance, which are popular evaluation metrics in the tasks of explicit rating commendation [54] and click-through rate prediction [55].

Equation (14) shows how to calculate RMSE.

(14) $$\begin{array}{c} L_{rmse}=\sqrt{\frac{1}{N}\underset{x\in X}{\sum }{\left(\hat{y}\left(x\right)-y\left(x\right)\right)}^{2},} \end{array}$$

where *X* represents the set of instances for testing, *N* is the number of instances, and $\hat{y}\left(x\right)$ and *y*(*x*) represent the predicted value and the ground-truth label of a instance *x*. A lower RMSE score indicates a better performance.

AUC is insensitive to the classification threshold and the positive ratio. AUC's upper bound is 1, and a larger value indicates a better performance. It reflects the sorting quality of the model.

Accuracy is the proportion of the samples that are predicted correctly. A larger value indicates a better performance.

In addition, we use the number of trainable parameters (Param#) to measure the complexity of different models and the training efficiency. If a model has a smaller number of parameters, the training time will cost less.

### 5.3. Implementation Environment

We develop the RFM model by using *Python* programming language, and Table 1 demonstrates the specifications of the environment in which the model was trained.

The article "Retrieval-Based Factorization Machines for Human Click Behavior Prediction" was published in 2022. Journal: Comput Intell Neurosci.

### 5.4. Baselines

We compare RFM with the following competitive methods that are designed for sparse data and CTR prediction in recommender systems.

- FM [5]: FM has shown a good performance for personalized recommendation and context-aware prediction, and it can effectively capture second-order feature interaction information. This is the infrastructure of many deep neural network models. We use the official *C*++ implementation (https://www.libfm.org/) for FM.
- HOFM [7]: This is the enhanced version of FM, which can capture high-order feature interaction information. We use the TensorFlow implementation of the high-order factorization machines.
- Wide&Deep [13]: This model consists of wide component and deep component. The wide component is a linear regression model, and the deep component first concatenates embedding vectors and is followed by an MLP [13] to model feature interactions.
- DeepCross [14]: This model concatenates embedding vectors, followed by a multilayered residual network. With the residual structure, the network can prevent gradient explosion and vanishing problem when the network deepens.
- DeepFM [15]: This model consists of one FM component and one deep component. It combines the power of factorization machines and deep learning to emphasize both low- and high-order feature interactions. Two components share the embedding parameters.
- HoAFM [30]: It uses a cross interaction layer to update a feature's representation by aggregating other cooccurred features and performs a bit-wise attention mechanism on the granularity of dimensions.
- PIN [28]: This method extends FM with kernel product methods to learn field-aware feature interactions and adopts a feature extractor to explore feature interactions to tackle the insensitive gradient issue.

### 5.5. Performance Comparison

Based on our investigation about parameters in the validation set, we set the default values of parameters in our RFM method. We set the embedding size *d* to 256 and the factor *β* to 1 by default in three datasets. The default value of the similarity threshold *r* in Frappe and MovieLens is 0.8, and it is 0.2 in Criteo. The top-*t* values are set as 6, 1, and 11 by default in the datasets of Frappe, MovieLens, and Criteo, respectively. The default value of the region number is 2 in Frappe and MovieLens, and it is 2^6^ in Criteo. We will demonstrate how to obtain those values in Section 5.7.

We set the initial learning rate as 0.01 and use Adagrad [56] as the model optimizer for RFM since Adagrad can adapt the learning rate during the training phase and ease the work of assigning a proper learning rate. For the other methods or models, we use the default learning rate configuration referred in their source codes or their articles.

The article "Retrieval-Based Factorization Machines for Human Click Behavior Prediction" was published in 2022. Journal: Comput Intell Neurosci.

We compare the performance of our RFM method and different baselines.  Table 2 summarizes the performance and the scale of trainable parameters obtained on embedding size 256.

According to Table 2, we have the following observations:

- RFM has the same scale of trainable parameters as FM. However, RFM performs better than FM by a 7.8%, 7.0%, and 1.6% average improvement in RMSE, AUC, and accuracy separately. This demonstrates the effectiveness of neighbor-based local information which enhances the original FM.
- HOFM uses a separated set of embeddings to model high-order feature interactions and achieves better performance than FM in the dataset of MovieLens and Criteo. However, the performance of HOFM is worse than that of FM in the dataset of Frappe. The reason is probably that although the high-order (more than 2) feature interactions can provide useful information, they also introduce noisy information simultaneously. Also, HOFM doubles the scale of parameters and incurs more training overhead.
- Wide&Deep and DeepCross take the feature embedding (Section 3.1) as the input of deep neural networks, which may miss the second-order feature interaction information if the embedding parameters are not initialized by pretrained FM model [16]. Thus, both of them almost have the worst performance. Furthermore, Wide&Deep and DeepCross have the most parameters.
- DeepFM can combine the knowledge from the feature embedding (Section 3.1) and second-order interactions embedding (Section 3.2) in the FM component, as well as high-order feature interaction from the deep component with sharing embedding parameters. Thus, generally, DeepFM has a good performance in the three datasets. However, sometimes, it performs poorly especially for the metric of RMSE in the MovieLens dataset, because MovieLens has only three fields and DeepFM may not capture enough useful feature interaction information. Besides, the deep component of DeepFM will lead to more training parameters and decreases the efficiency.
- HoAFM captures the high-order feature interactions in an explicit manner with the attentive FM, which is comparable to our RFM in the metric of AUC and accuracy for the dataset of MovieLens, but has a worse performance in other datasets.
- PIN obtains a good performance in the dataset of Criteo but performs poorly in the datasets of Frappe and MovieLens, which shows that sometimes the adaptive embeddings learned by the kernel product may be not effective.

The article "Retrieval-Based Factorization Machines for Human Click Behavior Prediction" was published in 2022. Journal: Comput Intell Neurosci.

Overall, our proposed RFM model achieves the best performance among these models in RMSE and AUC due to the enhancement of neighbor-based local information. RFM also has the same number of parameters with FM, which can achieve the best training efficiency.

### 5.6. The Effectiveness of Local Information

We take four examples from the testing sets to qualitatively analyze the effectiveness of neighbor-based local information in our approach.  Table 3 shows the four examples. In addition, we also show the percentages of testing samples where neighbors correct or worsen the output of FM for the three datasets in Table 4.

In Table 3, the first column is the ground-truth label of the given samples, and the second column is the original FM output of ${\hat{y}}_{g}\left(x\right)$. The third column represents the similarities between given samples from testing sets and their corresponding neighbors retrieved from the training set. The forth column is labels of neighbors. The last column is the final output by fusing the local knowledge and the original FM output. Obviously, the original FM outputs ${\hat{y}}_{g}\left(x\right)$ deviates from the true labels for the four examples, which means that the global knowledge learned by FM cannot model the click behavior correctly for these four examples. However, the neighbors from the training set, whose similarities are more than 0.8 (in the third column), can provide useful local knowledge with correct labels (as shown in the fourth column). Then, we use such local knowledge to correct the original FM output ${\hat{y}}_{g}\left(x\right)$ and obtain the final results (as shown in the last column). Intuitively, in the real scenario, original FM may predict that a user would not like to click one item because most of users in the training set dislike to click. But several other users who have similar characteristics to the user clicked the item, and the user also intends to click it with a high probability. In this way, the neighbor-based local information can represent the personal and preference knowledge and is effective to enhance the FM model.

Besides, we further record the percentages of three types of results from the testing sets, as shown in Table 4. The keywords “Better” and “Worse” mean that the fusion result is better or worse than ${\hat{y}}_{g}\left(x\right)$, and the symbol “Equal” represents that the fusion result is the same as ${\hat{y}}_{g}\left(x\right)$. We can see that RFM corrects most of the mistakes of ${\hat{y}}_{g}\left(x\right)$ in the testing sets and has a small negative impact at the same time. In the datasets of Frappe and MovieLens, the percentages of the worse cases are much smaller. In Criteo, the percentage of the worse cases is relatively higher than the other two datasets. However, the degree of positive cases (better, 63.17%) is much bigger than that of negative ones (worse, 35.87%). Therefore, RFM enhances the overall performance of FM in Criteo. The percentages of three types of results further illustrate that the neighbor-based local information captured by RFM is effective.

The article "Retrieval-Based Factorization Machines for Human Click Behavior Prediction" was published in 2022. Journal: Comput Intell Neurosci.

### 5.7. Hyperparameter Investigation

We explore the impact of four important hyperparameters including the number of regions *k*, the embedding size *d*, the number of similar samples *t*, and the similarity threshold *r*. Since the results of RMSE are similar to that of AUC, we only show RMSE in the following discussion. When investigating the effect of one hyperparameter, we remain other hyperparameters stable.

#### 5.7.1. The Number of Regions

We partition samples in the training set into multiple regions for the sake of efficiency and performance. It can not only accelerate the process of retrieving similar samples but also introduce the better region features. The former increases the efficiency, and the latter improves the effectiveness. We assign 2^*n*^ to the region number *k*, where *n* is from 0 to 7 with step size 1.

Figure 2 shows the influence of the region number on the performance of RFM for different datasets. We can see that the region partition can influence the performance, and it may improve the performance to some extent with the proper numbers of regions. Without region partition (i.e., *n* = 0 and the region number is 1), the model will retrieve neighbors by traversing all samples in the training set. We can observe that the performance is always not the best. When partitioning samples into multiple regions, each region has its own center vector for representing the common characteristics of samples in it. Figures 2(a) and 2(b) show that partitioning samples into two regions can have the best performance. Continuing to increase the region number will reduce the effectiveness, since dividing samples into too many regions may weaken the ability of a region to represent common characteristics of samples belonging to it. In Figure 2(c), we have the best performance when *n*=6, and the curve fluctuates frequently, which indicates that the characteristics of samples in Criteo are highly diverse. Intuitively, the retrieved similar samples may not be the most similar ones from the whole training set when the region number is more than 1 and probably decreases the performance. However, we can see that the region partition can improve the performance as well. That is because the clustering technique can reveal the intrinsic nature and regularity in the training set [46, 47], the most similar samples retrieved from the same region may contain more effective and generalizable information than those from the whole training set.

The article "Retrieval-Based Factorization Machines for Human Click Behavior Prediction" was published in 2022. Journal: Comput Intell Neurosci.

We also measure the efficiency of our RFM method for different region numbers. In Figure 3, we show the average prediction time (APT) for different region numbers, where APT is the average time to predict one sample in the testing set. For clarity, we take the natural logarithm of APT. As shown in Figure 3, the increase of the region number reduces APT roughly in a linear relationship, since the region partition can decrease the target samples for the retrieval of neighbors by the rate of the region number. If the region number keeps the same, generally, the APT depends on the sizes of the training sets in different datasets. For example, the size of Movielens dataset is the largest, and then, it needs more time to retrieve neighbors than the other two datasets. When the region's number is more than 2^5^, the APT of Criteo is less than that of Frappe, which is probably because different regions have different numbers of samples. In Criteo, the number of samples in the most similar region is smaller than those in Frappe, although it has more samples in the whole training set.

In summary, when considering the performance and prediction efficiency together, we can find the best choice of the region number that has a good trade-off between the performance and efficiency for one specific dataset. For example, we can choose *n*=6 as the best region partition for the Criteo dataset since it has the best performance with much high prediction efficiency.

#### 5.7.2. Embedding Size

The size of second-order feature interaction embedding may have an impact on the performance. As shown in Figure 4, we evaluate our RFM model and baselines in the Frappe dataset with different embedding sizes. For highlighting the sensitivity, we set a small step by 16 and show a small range of embedding sizes around 256 when RMSE changes. We find that RFM achieves the best performance compared to other methods for all experimental embedding sizes. Among them, when the embedding size is 256, RFM can have the best performance. We only show the RMSE for different embedding sizes in the Frappe dataset since the other two datasets have the similar trend.

#### 5.7.3. Top-*t* Similar Neighbors

The hyperparameter *t* determines the number of neighbors as the local information for fusion.  Figure 5 shows the RMSE of our model with regard to different top-*t* values.

As shown in Figure 5, the impact of top-*t* values on different datasets is different. The curve in Figure 5(a) is overall convex and local oscillating. Too small *t* cannot introduce enough local knowledge from neighbors, and too large *t* may introduce noisy neighbors. Then, we have Top-6 as an optimal value. Figure 5(b) shows that RMSE increases with the rise of top-*t*. This is because the number of fields in Movielens is only three, and neighbors contain less feature interaction information. When the number of neighbors increases, it may introduce more noisy data. By contrast, RMSE decreases with the rise of top-*t* in Figure 5(c), since the number of fields in Criteo is the most, and neighbors contain the richest and useful interaction information for the following fusion. The curves in Figures 5(b) and 5(c) become horizontal near the end due to the limitation introduced by the similarity threshold.

The article "Retrieval-Based Factorization Machines for Human Click Behavior Prediction" was published in 2022. Journal: Comput Intell Neurosci.

#### 5.7.4. The Similarity Threshold

The similarity threshold *r* is a key hyperparameter to filter out noisy neighbors. We investigate the influence of *r* on RMSE.  Figure 6 shows the result.

As shown in Figure 6, if the similarity threshold is too low, it will introduce more noisy data and decrease the effectiveness of our model. If the similarity threshold is too high, it will filter out some valuable knowledge and decrease the effectiveness as well. In Frappe and Movielens, 0.8 is the best similarity threshold, which has a good trade-off between filtering out noisy data and introducing valuable knowledge. The RMSEs before 0.8 are stable since we always select the same top-*t* neighbors. For the curve of Criteo, 0.2 is the best similarity threshold since the sample similarities are relatively small.

## 6. Conclusion

How to predict click-through rate (CTR) accurately is an important problem in many recommendation scenarios. In this work, we proposed a novel solution called retrieval-based factorization machine (RFM), which aims to predict CTR by combining global knowledge learned from the FM model with the neighbor-based local information. We conducted experiments on three public datasets to evaluate RFM, and the experimental results show that our RFM model outperformed existing models with a simple and efficient architecture. The results also indicate that using local information properly can enhance the overall performance of CTR-predicting tasks.

More generally, the idea of fusing global and local information in this paper can be applied in other domains, including some dense data tasks. There are two interesting directions for the future study. One is exploring strategies to retrieve effective neighbors and filter out noisy data more efficiently and accurately. The other is how to combine the local information with the original FM model better to predict human click behavior more effectively.

The article "Retrieval-Based Factorization Machines for Human Click Behavior Prediction" was published in 2022. Journal: Comput Intell Neurosci.

## Figures and Tables

**Figure 1:** The architecture of RFM.

**Figure 2:** RMSE for different region numbers.

**Figure 3:** Average prediction time for different region numbers.

**Figure 4:** RMSE for different embedding sizes.

**Figure 5:** RMSE for different top-t values.

**Figure 6:** RMSE for different similarity thresholds.

**Algorithm 1:** The algorithm of neighbor retrieval.

**Table 1:** Details of the implementation environment.

Environment	Specifications
Operating system	Ubuntu 20.04.5 LTS
Processor	Intel (R) xeon (R) silver 4116 CPU
Architecture	64-Bit
Memory	128 GB
GPU	NVIDIA V100 PCIe 32 GB
Programming language	*Python*
Framework	Tensorflow
Main libraries used	Pandas, numpy, sys, os

**Table 2:** RMSE, AUC, accuracy, and number of parameters for different models. The symbol *M* means “million.”

Model	Frappe				MovieLens				Criteo			
	RMSE	AUC	Accuracy (%)	Param#	RMSE	AUC	Accuracy (%)	Param#	RMSE	AUC	Accuracy(%)	Param#
FM	0.3452	0.9829	96.32	1.38 M	0.4735	0.9512	91.10	23.24 M	0.4679	0.6051	74.20	12.43 M
HOFM	0.3331	0.9218	95.53	2.76 M	0.4636	0.9582	91.47	46.40 M	0.4637	0.6505	75.12	24.86 M
Wide&Deep	0.3661	0.9720	96.27	4.59 M	0.5313	0.9341	85.04	24.71 M	0.4703	0.6371	72.96	23.58 M
DeepCross	0.4071	0.9660	95.00	8.95 M	0.5130	0.9352	87.90	29.01 M	0.4671	0.6881	74.93	35.15 M
DeepFM	0.3305	0.9815	96.82	4.15 M	0.4812	0.9591	91.89	24.58 M	0.4648	0.6671	75.27	27.33 M
HoAFM	0.3466	0.9829	97.02	1.54 M	0.4518	**0.9694**	**93.27**	23.37 M	0.4255	0.7201	76.38	13.82 M
PIN	0.3729	0.9707	96.35	2.10 M	0.5207	0.9424	91.09	23.29 M	0.4221	0.7191	76.30	49.55 M
**RFM**	**0.3225**	**0.9832**	**97.05**	**1.38 M**	**0.4509**	0.9611	93.24	**23.24 M**	**0.4113**	**0.7262**	**76.40**	**12.43 M**

**Table 3:** The effectiveness of neighbor-based local information.

Label	${\hat{y}}_{g}\left(x\right)$	Similarities	*Y*	Fusion
−1.0	0.0483	[0.8177, 0.8064, 0.8060, 0.8048, 0.8008]	[−1.0, −1.0, −1.0, −1.0, −1.0]	−0.7918
1.0	−0.0369	[0.8462, 0.8191, 0.8126, 0.8125, 0.8117]	[1.0, 1.0, 1.0, 1.0, 1.0, 1.0]	0.7967
1.0	−0.0125	[0.8369, 0.8358, 0.8347, 0.8346, 0.8343]	[1.0, 1.0, 1.0, 1.0, 1.0, 1.0]	0.8044
1.0	−0.0128	[0.8089, 0.8074, 0.8055, 0.8053, 0.8049]	[1.0, 1.0, 1.0, 1.0, 1.0, 1.0]	0.7987

**Table 4:** The percentage of three types of results.

	Better (%)	Equal (%)	Worse (%)
Frappe	63.96	34.86	1.18
MovieLens	76.86	18.04	5.10
Criteo	63.17	0.96	35.87

## Data Availability

The datasets used in this study are included within the article.
